The article "A Methanol Extract of Brugmansia arborea Affects the Reinforcing and Motor Effects of Morphine and Cocaine in Mice" was published in 2013. Journal: Evid Based Complement Alternat Med.

# A Methanol Extract of *Brugmansia arborea* Affects the Reinforcing and Motor Effects of Morphine and Cocaine in Mice

**DOI:** 10.1155/2013/482976

**Published:** 2013-03-07

**Authors:** Antonio Bracci, Manuel Daza-Losada, Maria Aguilar, Vincenzo De Feo, José Miñarro, Marta Rodríguez-Arias

**Affiliations:** ^1^Department of Pharmacy, University of Salerno, Via Ponte don Melillo, Salerno, 84084 Fisciano, Italy; ^2^Unidad de Investigación Psicobiología de las Drogodependencias, Departamento de Psicobiología, Facultad de Psicología, Universitat de Valencia, 46010 Valencia, Spain

## Abstract

Previous reports have shown that several of the effects of morphine, including the development of tolerance and physical withdrawal symptoms, are reduced by extracts of *Brugmansia arborea* (L.) Lagerheim (Solanaceae) (*B. arborea*). In the present study we evaluate the action of the methanol extract of *B. arborea* (7.5–60 mg/kg) on the motor and reinforcing effects of morphine (20 and 40 mg/kg) and cocaine (25 mg/kg) using the conditioned place preference (CPP) procedure. At the doses employed, *B. arborea* did not affect motor activity or induce any effect on CPP. The extract partially counteracted morphine-induced motor activity and completely blocked the CPP induced by 20 mg/kg morphine. On the other hand, *B. arborea* blocked cocaine-induced hyperactivity but did not block cocaine-induced CPP. Reinstatement of extinguished preference with a priming dose of morphine or cocaine was also inhibited by *B. arborea*. The complex mechanism of action of *B. arborea*, which affects the dopaminergic and the cholinergic systems, seems to provide a neurobiological substrate for the effects observed. Considered as a whole, these results point to *B. arborea* as a useful tool for the treatment of morphine or cocaine abuse.

## 1. Introduction 

Drug addiction is a chronically relapsing disorder characterized by a compulsion to seek and consume a substance, loss of control in limiting intake, and emergence of a negative emotional state when access to the drug is prevented [1]. A classification of the major classes of addictive drugs reveals that cocaine is clearly among the most dangerous, since both its addictive properties and capacity for physical harm are high, with only heroin and alcohol being considered as a greater threat [2, 3]. Although there are several pharmacological approaches approved for the treatment of opiate addiction, their partial effectiveness makes the search for new tools vital. Currently, there is no US Food and Drug Administration-approved medication for the treatment of cocaine addiction, and behavioral therapies alone demonstrate limited efficacy.

*Brugmansia arborea* (L.) Lagerheim is a solanaceous shrub native to South America and widely cultivated in Europe as an ornamental species. In Peru, this plant is employed by shamans in ritualistic ceremonies and for its anti-inflammatory, analgesic, vulnerary, decongestant, and antispasmodic properties, particularly in the treatment of rheumatic conditions [4]. Previous phytochemical studies have identified active components of the plant such as the tropane alkaloids hyoscine [5], atropine, norhyoscine, and scopolamine [6]. Methanol and water extracts of *B. arborea* have demonstrated affinity for 5-HT1A, 5-HT2A, 5-HT2C, D1, D2, *α*1, and *α*2 receptors in binding assays [7, 8], with a maximum affinity for D1 and D2 dopaminergic receptors.

Few pharmacological studies have been published about this plant. In one report, extracts, chromatographic fractions, and pure alkaloids from the species exerted an inhibitory activity on the contraction of isolated guinea pig ileum induced both electrically and by acetylcholine and on spasmolytic activity in vitro [9], thus indicating an anticholinergic activity. The three pure tropane alkaloids obtained from *B. arborea* were found to undermine symptoms in a concentration-dependent manner in an in vitro model of morphine withdrawal [10]. Moreover, in a recent report, *B. arborea* has been shown to reduce the expression of morphine tolerance and the development and expression of morphine dependence [11]. 

The aim of the present study was to use the conditioned place preference (CPP) procedure to assess whether or not the methanol extract of *B. arborea* can block the motor and reinforcing effects of morphine and cocaine. The CPP paradigm has been widely used to study the conditioned rewarding effects of addictive drugs, since contextual stimuli can acquire secondary appetitive properties (conditioned rewarding effects) when paired with a primary reinforcer, thereby increasing abuse liability [12]. In this paradigm, the conditioned rewarding properties of drugs are evaluated by pairing their effects with initially neutral cues, such as the compartment of an apparatus. The CPP test can be performed in a drug-free state, enabling the appetitive value of drug- associated contextual stimuli to be assessed while avoiding the confounding influence of consummatory variables. If, after conditioning, the animals spend more time in the compartment associated with the drug, it is assumed that the drug produces CPP. 

Drug addiction is a chronic, recurrent brain disease characterized by relapse [13]. The high rate of relapse to drug use after detoxification is a major clinical problem and constitutes the primary challenge to the treatment of drug abuse. In laboratory animals, it is possible to measure relapse when, following the acquisition and subsequent extinction of a particular behavioral response, the animal reinitiates this response, which is referred to as reinstatement [14]. There is a reinstatement model based on the CPP procedure that is employed to study relapse to drug abuse. The CPP induced by drugs of abuse can be extinguished and reinstated by drug priming [15].

## 2. Materials and Methods

### 2.1. Animals

A total of 228 male mice of the OF1 strain were acquired commercially from Charles River (Barcelona, Spain) at 42 days of age. They were housed in groups of four in plastic cages (25 × 25 × 14.5 cm) for 8 days prior to the initiation of experiments, under the following conditions: constant temperature (21 ± 2°C), a reversed light schedule (white lights on: 19.30–07.30 hours), and food and water available ad libitum, except during behavioral tests. Animals were handled on two consecutive days before the preconditioning (Pre-C) phase in order to reduce their stress levels in response to experimental manipulation. Procedures involving mice and their care were conducted in compliance with national, regional, and local laws and regulations, which are in accordance with the European Communities Council Directives (86/609/EEC, November 24, 1986). 

### 2.2. Plant Material, Extraction, Separation, and Identification

Aerial parts of *B. arborea* were collected in March 2008 in Conca dei Marini (Salerno, Italy). The plant was identified by Dr. V. de Feo. A voucher specimen of the plant (labeled as DF/2010/246) is stored at the herbarium of the Faculty of Pharmacy, University of Salerno. One kilogram of leaves and flowers of *B. arborea* were oven-dried at 40°C and powdered. The powder was extracted with methanol at room temperature for two days. The extract was concentrated in vacuo, which resulted in 32 g of residue. Aliquots of the extract of 3.5 g were purified on a Sephadex LH 20 column eluted with MeOH. Fractions were combined in 15 major fractions on the basis of their chemical similarity, as revealed by thin layer chromatography (TLC). Fractions 3 and 4, which both contained alkaloids, were purified by RF-HPLC. Pure apotropine (144.7 mg) was obtained from fraction 3 through purification using a C18 ì-Bondapak column under the following conditions: flow rate of 2.0 mL/min; eluent MeOH : H_2_O, 7 : 3. Atropine (152 mg) and 3á-tigloyl-oxitropane (212.3 mg) were obtained from fraction 4 through purification by RF-HPL using a C18 ì-Bondapak column under the following conditions: flow rate 2.0 mL/min; eluent MeOH : H_2_O, 6 : 4,. Pure compounds were identified by accurate NMR analyses and by comparing their spectral data with data available in the literature [16, 17].

### 2.3. Drug Administration

Doses of 7.5, 15, 30, and 60 mg/kg of *B. arborea* (crude methanol extract, B) were dissolved in water and immediately injected intraperitoneally (i.p.). Animals were also injected (i.p.) with 10 or 20 mg/kg of morphine (Laboratorios Sigma-Aldrich Química, Madrid, Spain) or 25 mg/kg of cocaine chlorhydrate (Laboratorio Alcaliber SA, Madrid, Spain). The drugs were diluted in physiological saline (NaCl 0.9%) at a constant volume (10 mL/kg). 

### 2.4. Motor Activity

Locomotor activity was measured automatically by an actimeter (CIBERTEC S.A., Spain) consisting of eight cages (33 × 15 × 13 cm), each with eight infrared lights located in a frame around the cage. Following 12 hours of adaptation to the actimeter, motor activity was recorded over a 6-hour period. Animals received one of the following treatments immediately before being placed in the actimeter: physiological saline (Sal, *n* = 8); 7.5 (B7.5, *n* = 8), 15 (B15, *n* = 7), 30 (B30, *n* = 7), or 60 (B40, *n* = 8) mg/kg of *B. arborea*; 40 mg/kg (M40, *n* = 8) of morphine; 40 mg/kg of morphine plus 7.5 (M40 + B7.5, *n* = 8), 15 (M40 + B15, *n* = 8), 30 (M40 + B30, *n* = 8), or 60 (M40 + B60, *n* = 8) mg/kg of *B. arborea* extract. For the cocaine study, the procedure was identical, only that the *B. arborea* extract was administered 1 hour before the drug. Animals were treated with 25 (C25, *n* = 11) mg/kg of cocaine, 25 mg/kg of cocaine plus 30 (C25 + B30, *n* = 12), or 60 (C25 + B60, *n* = 12) mg/kg of *B. arborea* extract. 

### 2.5. Conditioned Place Preference

The apparatus consisted of four identical Plexiglas place-conditioning boxes. Each of these boxes is comprised of two equally sized compartments (30.7 cm length × 31.5 cm width × 34.5 cm height) separated by a gray central area (13.8 cm length × 31.5 cm width × 34.5 cm height). The compartments have different colored walls (black versus white) and distinct floor textures (smooth in the black compartment and rough in the white one). Four infrared light beams in each compartment of the box and six in the central area allow the position of the animal and its crossings from one compartment to the other to be recorded. The equipment was controlled by an IBM PC computer using MONPRE 2Z software (CIBERTEC, SA, Spain).

This procedure, unbiased in terms of initial spontaneous preference, was performed as described previously [18]. In the first phase, referred to as preconditioning (Pre-C), mice were allowed to access to both compartments of the apparatus for 15 min (900 s) per day on 2 consecutive days. On day 3, the time spent in each compartment over a 900 s period was recorded. Animals showing a strong unconditioned aversion (less than 27% of the session time; i.e., 250 s) or preference (more than 73%; i.e., 650 s) for one compartment were eliminated from the rest of the study. In each group, half the animals received the drug or vehicle in one compartment and the other half in the other compartment. After assigning the compartments, an analysis of variance (ANOVA) revealed no significant differences between the time spent in the drug-paired and vehicle-paired compartments during the preconditioning phase. This is an important step in the experimental procedure that rules out any preference bias prior to conditioning. In the second phase (conditioning), which lasted 4 days, animals received an injection of physiological saline before being confined to the vehicle-paired compartment for 1 h. Following a further interval of 4 h, they received the corresponding dose of morphine, *B. arborea*, or both substances immediately before being confined to the drug-paired compartment for 1 h. During the third phase, known as postconditioning (Post-C), the guillotine door separating the two compartments was removed (day 8) and the time spent by the untreated mice in each compartment was recorded during a 900 s observation period. The difference in seconds between the time spent in the drug-paired compartment in the Post-C test and in the Pre-C phase is a measure of the degree of conditioning induced by the drug. If this difference is positive, then the drug has induced a preference for the drug-paired compartment, while the opposite indicates an aversion.

The animals were conditioned with 20 (M20, *n* = 9) or 40 (M40, *n* = 11) mg/kg of morphine; 30 (B30, *n* = 12) or 60 (B60, *n* = 11) mg/kg of *B. arborea* extract; 20 mg/kg of morphine plus 30 (M20 + B30, *n* = 10) or 60 (M20 + B60, *n* = 10) mg/kg of *B. arborea* extract; or 40 mg/kg of morphine plus 30 (M40 + B30, *n* = 11) or 60 (M40 + B60, *n* = 10) mg/kg of *B. arborea* extract.

For conditioning with cocaine, the procedure was similar, but during the conditioning phase animals were confined to each compartment for only 30 minutes. The *B. arborea* extract was always administered 60 minutes before the cocaine injection. The animals were conditioned with 25 (C25, *n* = 11) mg/kg of cocaine, 25 mg/kg of cocaine plus 30 (C25 + B30, *n* = 12), or 60 (C25 + B60, *n* = 12) mg/kg of *B. arborea* extract.

Conditioned groups underwent two extinction sessions per week in which animals were placed in the apparatus (without the guillotine doors separating the compartments) for 900 s until the time spent in the drug-paired compartment by each group was similar to that of Pre-C and different from that of the Post-C test. Extinction of CPP was always confirmed in a subsequent session of 24 hours after the last extinction session. The effects of the priming dose were evaluated 24 hours after confirmation of extinction. The reinstatement test was the same as that in Post-C (free ambulation for 900 s), except that animals were tested 15 minutes after administration of the respective dose of morphine or cocaine.

### 2.6. Statistical Analysis

The motor activity data were subjected to an analysis of variance (ANOVA) for repeated measures. A two-way ANOVA for locomotor activity was performed hourly for 6 hours, with two “between” subject variables—“dose of morphine,” with two levels (0 and 40 mg/kg), and “dose of *B. arborea,*” with five levels (0, 7.5, 15, 30 and 60 mg/kg)—and a “within” subject variable—“time,” with six levels. Bonferroni tests were employed to make post hoc comparisons. For the cocaine study, the same within variables were employed, but with only one “between” subject variable—treatment, with five levels (Sal, C25, C25 + B15, C25 + B30, and C25 + B60). 

In the CPP study, data relating to the time spent in the drug-paired compartment were analyzed using an analysis of variance (ANOVA) for repeated measures. A two-way ANOVA was performed for each conditioning, with a “between” subject variable—“treatment,” with eight levels (for the morphine data) or three levels (for the cocaine data)—and a “within” subject variable—“days,” with two levels: Pre-C and Post-C. Bonferroni tests were employed to make post hoc comparisons. Differences between the time spent by each group in the drug-paired compartment between each extinction session and reinstatement test were analyzed using paired Student's *t*-tests.

## 3. Results

The bioassay-oriented study of a methanol extract of *Brugmansia arborea* permitted the isolation of three tropane alkaloids: atropine, apoatropine, and 3*α*-tigloil-oxitropane. This is in accordance with the literature, in which there are reports that the genus *Brugmansia* contains this class of alkaloids [9, 19].

### 3.1. Morphine and *B. arborea*

#### 3.1.1. Motor Activity

Results over the six hours (Figures 1(a) and 1(b)) revealed that *B. arborea* did not modify motor activity; morphine produced a significant hyperactivity that the plant extract partially counteracted. The ANOVA showed that the M40, M40 + B7.5, and M40 + B15 groups were more active than the rest of the groups during the first four hours (F(4,66) = 3.664; *P* < 0.001). *B. arborea* counteracted morphine-induced hyperactivity, as the M40 + B60 group was more active than controls only during the second and third hours (*P* < 0.001), and the M40 + B30 group was most active than saline-treated counterparts only during the third hour (*P* < 0.05).

#### 3.1.2. Conditioned Place Preference

*B. arborea* has no reinforcing effects but is capable of blocking morphine-induced CPP (Figure 2). The ANOVA revealed that 40 mg/kg of morphine had reinforcing effects when administered alone or with *B. arborea*, as CPP (F(7,76) = 2.044; *P* < 0.05) was observed in all the groups conditioned with this dose of the drug (*P* < 0.05 for M40; *P* < 0.01 for M40 + B60; and *P* < 0.001 for M40 + B30). However, 20 mg/kg of morphine showed reinforcing effects only when administered alone or plus the lower dose of *B. arborea* (*P* < 0.05 for M20 and M20 + B30), and no CPP was observed in the M20 + B60 group. 

Among the groups that developed preference, the extinction process required 9 sessions in the M40 group, 29 sessions in the M40 + B30 group, 23 in the M40 + B60 group, and 4 in the M20 and M20 + B30 groups.

In the groups conditioned with 40 mg/kg of morphine, reinstatement of the extinguished preference after a priming dose of 20 mg/kg of morphine was observed only in the M40 group (*P* < 0.01). After 2 more extinction sessions, reinstatement was achieved with a dose of 10 mg/kg of morphine (*P* < 0.05). This preference was extinguished after 4 more extinction sessions. No reinstatement was observed after a priming dose of 5 mg/kg of morphine. 

Preference was reinstated in the M20 and M20 + B30 groups after a priming dose of 10 mg/kg of morphine (*P* < 0.01). Following 16 sessions, preference was not reinstated in the M20 group with a priming dose of 5 mg/kg of morphine. After 3 extinction sessions preference was reinstated in the M20 + B30 group with 5 mg/kg of morphine (*P* < 0.01). Following 2 more extinction sessions, no reinstatement was observed with a priming dose of 2.5 mg/kg of morphine. 

### 3.2. Cocaine and *B. arborea*

#### 3.2.1. Motor Activity

Results for the six-hour period (Figure 3) revealed that *B. arborea* blocked cocaine-induced hyperactivity. The ANOVA revealed higher activity in the group treated only with cocaine (F(3,27) = 25.391; *P* < 0.001) than in the Sal, C25 + B30, and C25 + B60 groups (*P* < 0.001) during the first four hours. In addition, levels of activity in the C25 + B30 group (F(5,135) = 7.064; *P* < 0.001) were higher than among saline-treated animals during the first hour (*P* < 0.001).

#### 3.2.2. Conditioned Place Preference

Although *B. arborea* did not block the reinforcing effects of cocaine, the higher dose impeded reinstatement of the extinguished preference. The ANOVA (Figure 4) revealed that all the groups developed CPP (F(1,36) = 51.820; *P* < 0.001) and spent more time in the drug-paired compartment on Post-C day (*P* < 0.001) than on Pre-C day. Preference was extinguished in the C25 group in 17 sessions, in the C25 + B60 group in 19 sessions, and in the C25 + B30 group in 5 sessions. Once preference was extinguished, CPP was reinstated in the C25 group with a priming dose of 12.5 mg/kg of cocaine (*P* < 0.001). A 6.25 mg/kg dose of cocaine did not restore the extinguished preference in this group after five extinction sessions (Figure 4). The extinguished preference was not reinstated in the C25 + B60 group with 12.5 mg/kg of cocaine, while the same dose reinstated CPP in the C25 + B30 group (*P* < 0.001). However, after 13 further extinction sessions, the extinguished preference was not reinstated with 6.25 mg/kg of cocaine.

## 4. Discussion 

Our results show that a methanol extract of *B. arborea* diminishes the reinforcing and motor effects of morphine and cocaine. At doses that did not modify motor activity or induce motivational effects, the *B. arborea* extract blocked the CPP induced by 20 mg/kg of morphine and counteract cocaine-induced hyperactivity in a dose-dependent manner. Although none of the doses of *B. arborea* employed in our study were capable of blocking cocaine-induced CPP, the highest one impeded priming-induced reinstatement of the preference. 

At the doses we assayed, the *B. arborea* extract did not exert any motor effect, but did block morphine-induced hyperactivity during the first two hours when administered in an intermediate dose (15 mg/kg). Surprisingly, the highest dose (60 mg/kg) exerted a lesser effect, counteracting morphine-induced hyperactivity only during the first hour. Given that *B. arborea* and morphine were administered at the same time, it is possible that the short-lived effects of the former were due to the fact that it has a shorter period of action than the latter, although the results of the second experiment somewhat challenge this explanation. As occurred in a previous study published by our group, cocaine induced a hyperactivity that lasted 4 hours [20], but this effect was counteracted during the whole recording time by *B. arborea* at doses of 30 and 60 mg/kg. In this case, the plant was administered 1 hour before cocaine due to the immediate effect that the latter exerts.

At the doses studied, *B. arborea* extracts did not induce CPP or conditioned place aversion (30 and 60 mg/kg), which rules out any motivational effect. In line with previous reports, 20 and 40 mg/kg of morphine induced a strong CPP [18] and preference was reinstated after extinction by a priming dose of morphine (20 and 10 mg/kg) [21]. Administration of the highest dose of *B. arborea* during the acquisition phase of conditioning blocked the CPP induced by 20 mg/kg of morphine. Although the CPP induced by 40 mg/kg of morphine was not blocked by administration of *B. arborea*, the extinguished preference was not reinstated in these groups. These results suggest that preference for this high dose of morphine developed during the acquisition phase, although the strength of the conditioning was diminished by coadministration of *B. arborea*, which resulted in a lack of reinstatement. One factor to take into consideration is the longer time required for extinction to be achieved in these groups. Animals conditioned with 40 mg/kg of morphine plus any of the doses of *B. arborea* required twice as long for the preference to be extinguished than those conditioned with only 40 mg/kg of morphine, which means that the likelihood of preference being reinstated is lesser. In this way, our results show that the *B. arborea* extract employed in the experiments is capable of blocking morphine-induced CPP and reinstatement of an extinguished preference.

None of the doses of *B. arborea* employed was capable of blocking a cocaine-induced CPP. However, animals conditioned with cocaine plus the highest dose of *B. arborea* did not show reinstatement after preference had been extinguished, which was probably a result of a weaker conditioning due to the coadministration of the two substances. In these animals, the time required to achieve extinction was similar to that in the group treated only with cocaine.

Our results demonstrate that *B. arborea* modifies the reinforcing and motor effects of morphine and cocaine. It is well known that mesolimbic dopaminergic neurons are implicated in the increase in locomotor activity induced by opioids and cocaine [22]. Equally, it is generally accepted that the dopamine mesolimbic system is critical to the achievement of a morphine-induced CPP [18, 23]. The fact that *B. arborea* extract has shown affinity for D1 and D2 DA receptors in binding assays [7, 8] suggests that an antagonism of these receptors is at least partially responsible for the blockade of the effects of morphine and cocaine observed. The DA antagonism induced by *B. arborea* extracts could affect multiple processes (reward, motivation, learning, memory, discrimination, locomotion, etc.). DA antagonism can block reward but also impairs the associative learning necessary for the acquisition of place conditioning. Drug addiction can be considered as a disorder of DA-dependent associative learning [24], and the fact that CPP and the hyperactivity induced by morphine are blocked by *B. arborea* extract suggests that this plant undermines the development of opiate addiction. Another possible explanation for the results obtained is the strong anticholinergic activity reported for a methanol extract of *B. arborea* [9]. Recent evidence implicates muscarinic acetylcholine receptors in the behavioral effects of drugs of abuse such as morphine and cocaine. For example, the pharmacological antagonism of muscarinic receptors modulates morphine's analgesic and reinforcing effects and is associated with withdrawal syndrome [25, 26]. Furthermore, there is direct evidence that nicotinic receptors mediate morphine reward [27] and morphine-induced reinstatement [28]. Similarly, muscarinic antagonists can alter the locomotor and rewarding effects of cocaine [25, 29, 30]; for instance, cocaine-induced CPP is inhibited by antagonism of the M1 muscarinic receptor [25]. Cholinergic pathways interact with DA systems at all levels of the reward circuit. Together with acetylcholine input into DA cell bodies, cholinergic systems could play a vital role in gating the flow of information concerning the motivational value of stimuli through the mesolimbic system [31].

## 5. Conclusion

*B. arborea* has previously been shown to modify many of the effects of morphine, including tolerance and dependence [9]. The present results support and extend such findings, since decreases in the reinforcing and motor effects of morphine were observed following *B. arborea* administration. Moreover, for the first time, we can report that *B. arborea* mediates the effects of cocaine. The complex mechanism of action of *B. arborea*, which affects the dopaminergic and cholinergic systems, seems to be a neurobiological substrate for the effects observed. Considered as a whole, these results point to *B. arborea* as a useful tool for the treatment of morphine or cocaine abuse.

## Figures and Tables

**Figure 1:** Means (±SEM) of locomotor activity (over six hours) in photocell cuts from adult mice treated with (a) physiological saline (Sal), 7.5, 15, 30, or 60 mg/kg of *B. arborea* (B7.5, B15, B30, and B60), and 40 mg/kg of morphine (M40) or (b) 40 mg/kg of morphine plus 7.5, 15, 30, or 60 mg/kg of *B. arborea* (M40 + B7.5, M40 + B15, M40 + B30, or M40 + B60). Differences with respect to mice treated with saline *P < 0.05; **P < 0.001.

**Figure 2:** Effects of *B. arborea* on the acquisition and reinstatement of morphine-induced CPP. Mice were conditioned with 30 or 60 mg/kg of *B. arborea* (B30 and B60), 20 or 40 mg/kg of morphine (M20 and M40), or 20 or 40 mg/kg of morphine plus 30 or 60 mg/kg of *B. arborea* (M40 + B30, M40 + B60, M20 + B30, and M20 + B60). Bars represent mean (±standard error of the mean) time spent in the drug-paired compartment before conditioning session (white), after conditioning session (black), during the last extinction session (light gray), and during the reinstatement test (dark gray). After extinction of CPP, mice performed the reinstatement test 15 min after a priming injection of 50%, 25%, or 12.5% of the morphine dose employed for conditioning. ***P < 0.001; **P < 0.01; *P < 0.05, significant difference with respect to preconditioning values; ^++^ *P* < 0.01; ^+^ *P* < 0.05, significant difference with respect to the previous extinction values.

**Figure 3:** Means (±SEM) of locomotor activity (over six hours) in photocell cuts from adult mice treated with physiological saline (Sal), 25 mg/kg of cocaine (C25) or 25 mg/kg of cocaine plus 30, or 60 mg/kg of *B. arborea* (C25 + B30 or C25 + B60). Differences with respect to mice treated with saline, **P < 0.001.

**Figure 4:** Effects of *B. arborea* on the acquisition and reinstatement of cocaine-induced CPP. Mice were conditioned 25 mg/kg of cocaine (C25), alone or plus 30 or 60 mg/kg of *B. arborea* (C25 + B30, C25 + B60). Bars represent mean (±standard error of the mean) time spent in the drug-paired compartment before conditioning session (white), after conditioning session (black), during the last extinction session (light gray), and during the reinstatement test (dark gray). After extinction of CPP, mice performed the reinstatement test 15 min after a priming injection of 50% or 25% of the cocaine dose employed in conditioning.^  ∗∗∗^ *P* < 0.001, significant difference with respect to preconditioning values; ^+++^ *P* < 0.001, significant difference with respect to the previous extinction values.
